The article "Herbal Supplement Ameliorates Cardiac Hypertrophy in Rats with CCl4-Induced Liver Cirrhosis" was retracted in 2017. Reasons: duplicated images; original data or images not available; concerns about the data; concerns about the images.

# Herbal Supplement Ameliorates Cardiac Hypertrophy in Rats with CCl_4_-Induced Liver Cirrhosis

**DOI:** 10.1155/2012/139045

**Published:** 2012-11-06

**Authors:** Ping-Chun Li, Yung-Wei Chiu, Yueh-Min Lin, Cecilia Hsuan Day, Guang-Yuh Hwang, Peiying Pai, Fuu-Jen Tsai, Chang-Hai Tsai, Yu-Chun Kuo, Hsiao-Chuan Chang, Jer-Yuh Liu, Chih-Yang Huang

**Affiliations:** ^1^Division of Cardiovascular Surgery, China Medical University Hospital, Taichung 40402, Taiwan; ^2^Department of Life Science, Tunghai University, Taichung 40704, Taiwan; ^3^Emergency Department and Center of Hyperbaric Oxygen Therapy, Tungs' Taichung MetroHarbor Hospital, Taichung 43503, Taiwan; ^4^Institute of Medicine, Chung Shan Medical University, Taichung 40201, Taiwan; ^5^Department of Pathology, Changhua Christian Hospital, Changhua 50006, Taiwan; ^6^Department of Nursing, MeiHo University, Pingtung 91202, Taiwan; ^7^Division of Cardiology, China Medical University Hospital, Taichung 40402, Taiwan; ^8^Graduate Institute of Chinese Medical Science, China Medical University, Taichung 40402, Taiwan; ^9^Department of Healthcare Administration, Asia University, Taichung 41354, Taiwan; ^10^Graduate Institute of Basic Medical Science, China Medical University, Taichung 40402, Taiwan; ^11^Department of Biotechnology, Asia University, Taichung 41354, Taiwan; ^12^Center for Molecular Medicine, China Medical University Hospital, Taichung 40402, Taiwan; ^13^Graduate Institute of Cancer Biology, China Medical University, Taichung 40402, Taiwan; ^14^Department of Health and Nutrition Biotechnology, Asia University, Taichung 41354, Taiwan

## Abstract

We used the carbon tetrachloride (CCl_4_) induced liver cirrhosis model to test the molecular mechanism of action involved in cirrhosis-associated cardiac hypertrophy and the effectiveness of *Ocimum gratissimum* extract (OGE) and silymarin against cardiac hypertrophy. We treated male wistar rats with CCl_4_ and either OGE (0.02 g/kg B.W. or 0.04 g/kg B.W.) or silymarin (0.2 g/kg B.W.). Cardiac eccentric hypertrophy was induced by CCl_4_ along with cirrhosis and increased expression of cardiac hypertrophy related genes NFAT, TAGA4, and NBP, and the interleukin-6 (IL-6) signaling pathway related genes MEK5, ERK5, JAK, and STAT3. OGE or silymarin co-treatment attenuated CCl_4_-induced cardiac abnormalities, and lowered expression of genes which were elevated by this hepatotoxin. Our results suggest that the IL-6 signaling pathway may be related to CCl_4_-induced cardiac hypertrophy. OGE and silymarin were able to lower liver fibrosis, which reduces the chance of cardiac hypertrophy perhaps by lowering the expressions of IL-6 signaling pathway related genes. We conclude that treatment of cirrhosis using herbal supplements is a viable option for protecting cardiac tissues against cirrhosis-related cardiac hypertrophy.

## 1. Introduction

Patients with advanced cirrhosis have consistently been diagnosed with cardiac dysfunction under the condition of hyperdynamic circulation [1]. Increased cardiac output and reduced systemic vascular resistance are both signs of this condition [2–4]. Although cardiac dysfunction in patients with cirrhosis and potential clinical implications have long been known [5], little is understood regarding the molecular mechanism of action involved in cirrhosis-associated alteration in cardiac structure and function, especially cardiac hypertrophy.

Cirrhosis is known as a possible cause of portal vein constriction which may induce the activation of vasopressin, angiotensin II (Ang II), and the sympathetic nervous system [6]. Cardiac hypertrophy is induced by such direct mechanical wall stress as well as paracrine/autocrine factors such as Ang II, which in turn activates specific signaling pathways, for instance, mitogen-activated protein kinases (MAPKs) and calcineurin. These can cause cardiac hypertrophy and increase of related gene expressions, such as proto-oncogenes c-Fos and c-JUN, genes which encode atrial natriuretic peptide (ANP) and B-type natriuretic peptide (BNP), and structural genes *β*-myosin heavy chain (*β*-MHC) and skeletal *α*-actin [7]. Ang II is associated with increased plasma levels of proinflammatory cytokines such as interleukin-6 (IL-6) [8], which is an effective stimulator of the Janus kinase/signal transducer and activator of transcription (JAK/STAT) pathway in cardiac hypertrophy [7]. However, the role of these protein markers and transcriptional factors in cardiac hypertrophy and remodeling *in vivo* has not been examined in cirrhosis-associated hypertrophy. 

Carbon tetrachloride (CCl_4_) is frequently used to induce experimental cirrhosis in rats [9]. This model has recently been used to investigate the role of lipophilic bile acids and examine cardiac gene expression profiles in cirrhotic cardiomyopathy [10, 11]. Silymarin, a standardized extract of the *milk thistle* (*Silybum marianum *L. Gaertner), contains three biochemicals: silybin, silydianin, and silychristin and has a long tradition as a herbal remedy [12]. *Ocimum gratissimum* extract (OGE), a commonly used herb in folk medicine, is rich in antioxidants and possesses many therapeutic functions [13–21]. Both herbal extracts have been shown using the CCl_4_ model to inhibit liver cirrhosis [22]. Therefore the motive for this experiment is to use the CCl_4_-induced liver cirrhosis model to understand the molecular mechanism of action involved in cirrhosis-associated cardiac hypertrophy, as well as to test effectiveness of silymarin and OGE against cardiac damage and hypertrophy.

## 2. Materials and Methods

### 2.1. Preparation of OGE

Leaves of *Ocimum gratissimum *were harvested and washed with distilled water followed by homogenization with distilled water using polytron. The homogenate was incubated at 95°C for 1 hour (h) and then filtered through two layers of gauze. The filtrate was centrifuged at 20,000 g, 4°C for 15 minutes (min) to remove insoluble pellets and the supernatant (OGE) was thereafter collected, lyophilized, and stored at −20°C until use. The final extract (OGE) was composed of 11.1% polyphenol (including 0.03% catechins, 0.27% caffeic acid, 0.37% epicatechin, and 3.27% rutin). 

### 2.2. Animals and Treatment

Forty male wistar rats weighing 200–240 g were purchased from the National Animal Center and housed in conventional cages with free access to water and rodent chow at 20–22°C with a 12-hour light-dark cycle. All procedures involving laboratory animal use were in accordance with the guidelines of the Instituted Animal Care and Use Committee of Chung Shan Medical University (IACUC, CSMU) for the care and use of laboratory animals. The rats were divided evenly into five groups of 8 rats and treated intraperitoneally with CCl_4_ (8% CCl_4_/corn oil, 1 mL/kg body weight (BW) twice a week, Monday and Thursday) for 8 weeks, as described by Hernández-Muoz et al. [23], with some modifications. At the same time, the rats were treated with various dosages of OGE (0–0.04 g/kg BW), or silymarin orally (0.2 g/kg BW, four times a week, Tuesday, Wednesday, Friday, and Saturday) [24, 25]. The control rats were treated with corn oil (1 mL/kg BW) and fed a normal diet. At the end of the experiment, blood and heart were immediately obtained after the animals were sacrificed. 

### 2.3. Histological Examinations

The heart was fixed in 10% formalin, processed using routine histology procedures, embedded in paraffin, cut in 5 *μ*m sections, and mounted on a slide. The samples were stained with hematoxylin and eosin for histopathological examination. 

### 2.4. Preparation of Tissue Extract

All procedures were performed at 4°C. The heart samples were lysed by 30 strokes using a Kontes homogenizer at a ratio of 100 mg tissue/1 mL lysis buffer. The lysis buffer consisted of 50 mM Tris-HCl (pH 7.4), 2 mM EDTA, 2 mM EGTA, 150 mM NaCl, 1 mM PMSF, 10 *μ*g/mL leupeptin, 1 mM sodium orthovanadate, 1% (v/v) 2-mercaptoethanol, 1% (v/v) Nonidet P40, and 0.3% sodium deoxycholate. These homogenates were centrifuged at 100,000 g for 1 h at 4°C. The supernatant was stored at −70°C for Western blot assay.

### 2.5. Electrophoresis and Western Blot

Tissue extract samples were prepared as described above. Sodium do deco sulfate-polyacrylamide gel electrophoresis is carried out as described by Laemmli [26] using 10% polyacrylamide gels. After samples are electrophoresed at 140 V for 3.5 h, the gels are equilibrated for 15 min in 25 mM Tris-HCl, pH 8.3, containing 192 mM glycine and 20% (v/v) methanol. Electrophoresed proteins are transferred to nitrocellulose paper (Amersham, Hybond-C Extra Supported, 0.45 Micro) using Hoefer Scientific Instruments Transpher Units at 100 mA for 14 h. The nitrocellulose paper was incubated at room temperature for 2 h in blocking buffer containing 100 mM Tris-HCl, pH 7.5, 0.9% (w/v) NaCl, 0.1% (v/v) Tween 20, and 3% (v/v) fetal bovine serum. Antibodies BNP, phospho-GATA binding protein 4 (p-GATA4), nuclear factor of activated T cells (NFAT), mitogen-activated protein kinase kinase 5 (MEK5), extracellular signal-regulated protein kinase 5 (ERK5), phospho-extracellular signal-regulated protein kinase 5 (p-ERK5), phospho-Janus kinase (p-JAK), signal transducer and activator of transcription 3 (STAT3), *α*-tubulin purchased from Santa Cruz Biotechnology, Inc. (CA, USA), and IL-6 purchased from Abcam Inc. (MA, USA) are diluted to 1 : 2000 in antibody binding buffer containing 100 mM Tris-HCl, pH 7.5, 0.9% (w/v) NaCl, 0.1% (v/v) Tween 20, and 1% (v/v) fetal bovine serum. Incubations were performed at room temperature for 3.5 h. The immunoblots were washed three times in 50 mL blotting buffer for 10 min and then immersed for 1 h in the second antibody solution containing horseradish peroxidase goat anti-rabbit or anti-mouse IgG (Promega, WI, USA), which were diluted in binding buffer to 1000-fold, for various antibodies. After washing with blocking buffer, the membrane was visualized using chemiluminescence (Amersham Pharmacia Biotech, Piscataway, NJ, USA).

### 2.6. Statistical Analysis

The experimental results are expressed as the mean ± SE. Data were assessed using analysis of variance (ANOVA) followed by a Student-Newman-Keuls correction to adjust the significance level to avoid a type I error. Student's *t*-test was used in the comparison between groups. A *P* value less than 0.05 was considered statistically different. 

## 3. Results

### 3.1. Changes in Heart Weight of CCl_4_-Induced Cirrhosis-Associated Cardiac Hypertrophy

Throughout the experimental period of 8 weeks, there was no difference in body weight of rats within the 5 groups. At the end of the experiments when rat livers were measured, liver fibrosis was observed in the CCl_4_-treated group, as compared to the control group which was given olive oil. And for the groups treated with OGE or silymarin, a protective effect was observed: liver fibrosis was significantly ameliorated compared to the CCl_4_-treated group (data pending publication). In comparison, Table 1 shows that the whole heart weight (WHW), left ventricle weight (LVW), and their ratio to the body weight of the CCl_4_-treated group were significantly higher than the control group. For groups treated with 0.02 g/kg BW OGE and treated with 0.2 g/kg BW silymarin, weights of the heart remained equal to the control group. However, for the group treated with 0.04 g/kg BW OGE, the weight values had a less significant decrease compared to the CCl_4_-treated only group. 

### 3.2. Changes in Diameter and Thickness and Histological Structure of Left Heart Ventricle of CCl_4_-Induced Cirrhosis-Associated Cardiac Hypertrophy

The left ventricle diameter of the CCl_4_-treated group was significantly larger and the walls were moderately thicker than the control group (Figure 1 upper panel and Table 2), but a change of that scale in ventricle diameter was not present in the OGE and silymarin cotreated groups.

The left most picture in Figure 1 (lower panel) shows the appearance of a normal heart: one with a unified tissue pattern. However, hearts treated with CCl_4_ had clearly lost its tissue integrity, but such a change was clearly not observed in groups cotreated with 0.02 g/kg BW OGE and silymarin. 

### 3.3. The Expression of Cardiac Hypertrophy Related Genes in the Heart of CCl_4_-Treated Rats

The expression of cardiac hypertrophy related genes, such as BNP, p-GATA4, and NFAT4, were also tested [7]. Their figures were increased in the CCl_4_-treated group as compared to the control group (Figures 2 and 3). In the groups cotreated with 0.02 g/kg BW OGE or silymarin, the expression of BNP, p-GATA4, and NFAT returned to control level. The results of the 0.04 g/kg BW OGE-treated group were consistent with the above figures, in that their expressions were decreased, but not back to control levels.

### 3.4. The Expression of IL-6 Signaling Pathway Related Genes in the Heart of CCl_4_-Treated Rats

We wanted to test for IL-6 signaling pathways because studies have shown that cardiac hypertrophy can be attributed to IL-6 related cytokines [7]. Western blotting analysis shows that the expressions of IL-6, MEK5, ERK5, and p-ERK5 were increased in the CCl_4_-treated group as compared to the control group (Figure 4). In the groups cotreated with 0.02 g/kg BW OGE or silymarin, the expression of IL-6, MEK5, ERK5, and p-ERK5 returned to control level. The expressions were also lowered in the 0.04 g/kg BW OGE-treated group, but not back to the levels of the control group.

The expressions of other IL-6 signaling pathway genes, p-JAK and STAT3, were tested, the data shows that both their expressions were increased in the CCl_4_-treated group as compared to the control group (Figure 5). In the groups cotreated with 0.02 g/kg BW OGE or silymarin, the expressions of p-JAK and STAT3 returned to control levels, except for the 0.04 g/kg BW OGE group, which were lowered but not back to the control levels. This result is consistent with the data above.

## 4. Discussion

Numerous reports center on the involvement of IL-6 and the related cytokines in cardiac hypertrophy [7] as an inducer of downstream pathways. IL-6 is a typical cytokine which was found to have a potent hypertrophic effect on cardiomyocytes [27], as the overexpression of this cytokine has been linked to hypertrophic myocardium injury [28]. In the present study, our data showed that the expressions of IL-6 increased in CCl_4_-induced cirrhosis rats detected with occurrence of cardiac hypertrophy, which suggests that the cirrhosis-associated cardiac hypertrophy may be related with the IL-6 signaling pathway in the CCl_4_-treated rats.

IL-6 is involved in multiple intracellular signaling pathways, particularly the MEK5-ERK5 pathway [29–32], which plays a critical role in the induction of eccentric cardiac hypertrophy that can progress to dilated cardiomyopathy and sudden death [33, 34], and the JAK-STAT3 pathway, which promotes the increase of cell dimensions [35–37]. Since the experiments suggest a relationship between CCl_4_-induced cirrhosis-associated cardiac hypertrophy and IL-6, we decided to analyze the mechanism concerning OGE and silymarin and how it may inhibit cardiac hypertrophy through the inhibition of IL-6 extracellular signals. Western blotting analysis shows that the expressions of IL-6, MEK5, ERK5, and p-ERK5 were increased in the CCl_4_-treated groups as compared to the control (Figure 4) and were partially restored to control levels when cotreated with OGE or silymarin. Moreover, the expressions of p-JAK and STAT3 were increased in the CCl_4_-treated group (Figure 5) and restored by OGE or silymarin cotreatment, as in the above gene expressions. Taken together, these findings indicate that both the JAK-STAT3 and the MEK5-ERK5 pathways related genes were overexpressed by IL-6 expression in response to CCl_4_-induced cirrhosis-associated cardiac hypertrophy (Figure 6), which confirms the importance of the two pathways and also demonstrates that their overexpression may be reversed by OGE or silymarin treatment thus lowering liver cirrhosis and reducing the chance of cardiac hypertrophy. An interesting note is that silymarin, which has rarely been demonstrated to treat cardiac hypertrophy [38], suggests that some common elements between herbal preparations, such as their antioxidant properties, may be responsible for treatment against liver cirrhosis-induced cardiac damage.

Cardiac hypertrophy can be classified as physiological and pathological hypertrophy [7], with the physiological being a natural bodily response to maturation, pregnancy, and exercise, and the pathological being a response to pathological stress signals, such as inflammation, cardiac injury, or exposure to toxicity. In our study, we found that many genes was responded to cardiac hypertrophy by CCl_4_ induction, including MEK5, ERK5, JAK2, STAT3, NFAT3, GATA4, and fetal gene BNP, which are used as a pathological marker [39–42] (Figure 6). Since pathological hypertrophy is also associated with observable loss of tissue integrity, which we also found in CCl_4_-treated rats, this suggests that CCl_4_ induced cirrhosis-associated cardiac hypertrophy may belong to pathological hypertrophy and can also be explored further as a pathological model.

There is a peculiar phenomenon that a 0.02 g/kg BW dose of OGE had a significant inhibition effect on CCl_4_-induced cardiac hypertrophy and on the related gene expressions than a 0.04 g/kg BW dose. A possible explanation suggests that the saturation of the higher dose could have lowered the effectiveness of the treatment. 

## 5. Conclusions

In summary, CCl_4_-induced cirrhotic cardiac damage can occur through the IL-6 signaling pathway which leads to eventual cardiac hypertrophy. OGE and silymarin can protect cardiac cells from CCl_4_-induced damage possibly by inhibiting the expression of the IL-6 signaling pathway related genes. Moreover, we also found in further research that CCl_4_ induced cardiac damage can induce the FASL signaling pathway and the TGF-*β* signaling pathway, which may lead to cell apoptosis and eventual cardiac fibrosis (pending publication). It seems that multiple mechanisms are involved in the CCl_4_ induced cardiac damage. However, in the present study, we suggest that OGE and silymarin in the form of herbal supplements are a viable option for the protection of cardiac tissues against cirrhosis-related cardiac hypertrophy.

## Figures and Tables

**Figure 1:** Cardiac pathologic analysis in the heart of CCl_4_-treated rats. Herbs and CCl_4_ were given as described in Materials and Methods. The top panels show the heart of the macroscopic cross-section. The bottom panels show high magnification (×400) of tissue structure. LV: left heart ventricle; RV: right heart ventricle.

**Figure 2:** The expressions of BNP by Western blotting analysis (a) and quantitative analysis (b) in the heart of CCl_4_-treated rats. The individual severity rates in rats were expressed as mean ± SE, *n* = 8. *P < 0.05 as compared with control group. ^#^ *P* < 0.05 as compared with the CCl_4_-treated group.

**Figure 3:** The expressions of NFAT3 and phosphorylated-GATA4 by Western blotting analysis (a) and quantitative analysis (b) in the heart of CCl_4_-treated rats. The individual severity rates in rats were expressed as mean ± SE, *n* = 8, *P < 0.05 as compared with control group, and ^#^ *P* < 0.05 as compared with CCl_4_-treated group.

**Figure 4:** The expressions of IL6 and its downstream signaling proteins MEK5, ERK5, and phosphorylated-ERK5 by Western blotting analysis (a) and quantitative analysis (b) in the heart of CCl_4_-treated rats. The individual severity rates in rats were expressed as mean ± SE, *n* = 8, *P < 0.05 as compared with control group, and ^#^ *P* < 0.05 as compared with CCl_4_-treated group.

**Figure 5:** The expressions of JAK-Stat3 pathway by Western blotting analysis (a) and quantitative analysis (b) in the heart of CCl_4_-treated rats. The individual severity rates in rats were expressed as mean ± SE, *n* = 8. *P < 0.05 as compared with control group. ^#^ *P* < 0.05 as compared with CCl_4_-treated group.

**Figure 6:** The summary of the mechanism of CCl_4_-induced cirrhosis-associated cardiac hypertrophy. Our data demonstrated that *Ocimum gratissimum* and silymarin extracts attenuate cardiac cells from CCl_4_ induced damage possibly by lowering liver cirrhosis which reduces the chance of cardiac hypertrophy maybe via inhibiting IL-6 signaling pathway activation.

**Table 1:** Changes in body weight and organ weight of CCl_4_-induced cirrhosis-related cardiac hypertrophy.

	A^a^	B	C	D	E
	(*n* = 8)	(*n* = 8)	(*n* = 8)	(*n* = 8)	(*n* = 8)
BW (g)	425 ± 16.475	402 ± 8.920	385 ± 6.547	388 ± 10.823	420 ± 19.272
WHW (g)	1.041 ± 0.015	1.173 ± 0.031*	0.975 ± 0.023^#^	1.089 ± 0.026	1.023 ± 0.015^#^
LVW (g)	0.813 ± 0.010	0.898 ± 0.018*	0.745 ± 0.028^#^	0.777 ± 0.021	0.767 ± 0.023^#^
WHW/BW (%)	2.467 ± 0.095	2.918 ± 0.093*	2.535 ± 0.065^#^	2.813 ± 0.067	2.461 ± 0.101^#^
LVW/BW (%)	1.922 ± 0.050	2.233 ± 0.045*	1.933 ± 0.054^#^	2.190 ± 0.062	1.844 ± 0.085^#^
LVW/WHW (%)	0.781 ± 0.011	0.767 ± 0.012	0.764 ± 0.020	0.779 ± 0.015	0.751 ± 0.030

^a^ Group A is given olive oil and water, Group B is given CCl_4_ and water, Group C is given CCl_4_ and 0.02 g/kg of OGE, Group D is given CCl_4_ and 0.04 g/kg of OGE, and Group E is given CCl_4_ and 0.2 g/kg of silymarin. The individual severity rates in rats were expressed as mean ± SE. BW: body weight; WHW: whole heart weight; LVW: left ventricle weight. *Significant differences from Group A, *P* < 0.05. ^#^Significant differences from Group B, *P* < 0.05.

**Table 2:** Changes in diameter and thickness of left heart ventricle of CCl_4_-induced cirrhosis-related cardiac hypertrophy.

	A^a^	B	C	D	E
	(*n* = 8)	(*n* = 8)	(*n* = 8)	(*n* = 8)	(*n* = 8)
Diameter of LV (mm)	8.17 ± 0.00	10.67 ± 0.22*	8.50 ± 0.19^#^	9.33 ± 0.22^#^	8.83 ± 0.11^#^
Thickness of LV (mm)	3.83 ± 0.11	4.43 ± 0.15*	3.87 ± 0.12^#^	4.17 ± 0.11	3.83 ± 0.11^#^
Thickness/diameter (mm)	0.42 ± 0.01	0.42 ± 0.01	0.46 ± 0.02	0.45 ± 0.02	0.43 ± 0.01

^a^ Group A is given olive oil and water, Group B is given CCl_4_ and water, Group C is given CCl_4_ and 0.02 g/kg of OGE, Group D is given CCl_4_ and 0.04 g/kg of OGE, and Group E is given CCl_4_ and 0.2/kg g of silymarin. The individual severity rates in rats were expressed as mean ± SE. LV: left ventricle. *Significant differences from Group A, *P* < 0.05. ^#^Significant differences from Group B, *P* < 0.05.
